# Multispectral Image under Tissue Classification Algorithm in Screening of Cervical Cancer

**DOI:** 10.1155/2022/9048123

**Published:** 2022-01-07

**Authors:** Pei Wang, Shuwei Wang, Yuan Zhang, Xiaoyan Duan

**Affiliations:** ^1^Department of Gynaecology, Hebei Provincial People's Hospital, Shijiazhuang 050051, Hebei, China; ^2^Department of Gynaecology, Chengde Hospital of Traditional Chinese Medicine, Chengde 067000, Hebei, China

## Abstract

The objectives of this study were to improve the efficiency and accuracy of early clinical diagnosis of cervical cancer and to explore the application of tissue classification algorithm combined with multispectral imaging in screening of cervical cancer. 50 patients with suspected cervical cancer were selected. Firstly, the multispectral imaging technology was used to collect the multispectral images of the cervical tissues of 50 patients under the conventional white light waveband, the narrowband green light waveband, and the narrowband blue light waveband. Secondly, the collected multispectral images were fused, and then the tissue classification algorithm was used to segment the diseased area according to the difference between the cervical tissues without lesions and the cervical tissues with lesions. The difference in the contrast and other characteristics of the multiband spectrum fusion image would segment the diseased area, which was compared with the results of the disease examination. The average gradient, standard deviation (SD), and image entropy were adopted to evaluate the image quality, and the sensitivity and specificity were selected to evaluate the clinical application value of discussed method. The fused spectral image was compared with the image without lesions, it was found that there was a clear difference, and the fused multispectral image showed a contrast of 0.7549, which was also higher than that before fusion (0.4716), showing statistical difference (*P* < 0.05). The average gradient, SD, and image entropy of the multispectral image assisted by the tissue classification algorithm were 2.0765, 65.2579, and 4.974, respectively, showing statistical difference (*P* < 0.05). Compared with the three reported indicators, the values of the algorithm in this study were higher. The sensitivity and specificity of the multispectral image with the tissue classification algorithm were 85.3% and 70.8%, respectively, which were both greater than those of the image without the algorithm. It showed that the multispectral image assisted by tissue classification algorithm can effectively screen the cervical cancer and can quickly, efficiently, and safely segment the cervical tissue from the lesion area and the nonlesion area. The segmentation result was the same as that of the doctor's disease examination, indicating that it showed high clinical application value. This provided an effective reference for the clinical application of multispectral imaging technology assisted by tissue classification algorithm in the early screening and diagnosis of cervical cancer.

## 1. Introduction

Cervical cancer is a common malignant tumor in women. Its incidence ranks third in the world and ranks among the top three fatal gynecological tumors in most developing countries. According to a report from the World Health Organization (WHO), approximately 550,000 women worldwide become patients with new cases of cervical cancer each year, and more than half of these patients die of cervical cancer. As a developing country, China has more than 150,000 new patients with cervical cancer each year, of which more than 60,000 fatal cases accounting for more than 30% of new female patients with cervical cancer in the world. In recent years, the number of young female patients has gradually increased [1]. The site of cervical cancer is in the female cervix, and the cause is the growth and proliferation of abnormal cells in the female body. Early cervical cancer generally has no special differential symptoms, and late cervical cancer can develop into cervical cancer in situ and cervical invasive cancer [2]. Some countries under development and with scarce medical resources lack advanced medical resources and inspection equipment, so that women cannot get timely early screening and diagnosis, leading to cervical cancer gradually becoming the death killer of women.

The early diagnosis and identification methods of cervical cancer mainly include cell smear, colposcopy, and biopsy [3]. These examination methods have different shortcomings. For example, the cell smear method can easily lead to missed diagnosis of cancer cells because of the limited available cell smears; and the colposcopy method is mainly the result of the subjective judgment of the colposcopy doctor, so it is highly subjective and cannot make individualized diagnosis of patients. For female patients, the biopsy method needs to bear a physical and psychological burden, the test results are usually not available in a short time, and it is easy to delay the patient's treatment opportunity [4,5]. Cervical cancerous tissue will undergo physiological and pathological changes, which will cause optical changes in the tissue. Optical pathological diagnosis can avoid the above defects and has the characteristics of noninvasive and rapid. Especially, multispectral imaging technology has been widely used in recent years. Multispectral imaging technology is a new photoelectric detection technology. As an analysis tool, it has been widely used in many fields including biomedicine due to its unique technical advantages of both spectral detection and imaging. The biggest difference between multispectral imaging technology and ordinary imaging technology is that it converts black and white imaging or red, blue, and green imaging with low color accuracy into spectral imaging with higher color dimensions. A set of image sequences collected at different band positions are used to accurately record the “color” information of the marker sample and to obtain a high-resolution spectrum of each pixel in the image, instead of the three primary color images seen by the naked eye. With the assistance of multispectral fluorescence microscopes, quantum dots can achieve high accuracy and sensitive quantitative detection of molecular information, in situ and real-time co-imaging, and multimolecule co-imaging and interaction. Multispectral fluorescence imaging based on quantum dots can help improve tumor classification and predict tumor prognosis. Hu and Ma [6] used the snapshot multispectral narrowband imaging technology to accelerate the spectral image acquisition process, improve the gray-scale contrast between tissues of different disease levels, and realize the automatic classification of cervical tissue lesions with high frame rate.

In order to better screen for cervical cancer, it is necessary to identify and segment the image of the lesion. At present, the extraction of cervical cancer image lesions is generally performed by doctors for manual segmentation, which depends on the doctor's theoretical knowledge and experience, and is highly subjective. In addition, it is time-consuming and labor-intensive, more and more images need to be processed, and manual segmentation obviously cannot meet the demand. With the application of computer algorithms in medical imaging, the use of intelligent algorithms for automatic or semiautomatic segmentation of lesions can greatly reduce the workload of doctors. The tissue classification algorithm is through the aid of computer algorithms; all elements in the original image will be summarized into several clusters with different differences [7]. The elements in the cluster have similar elements, but there are big differences between clusters [8]. That is, after inputting the original feature map, it is a computer technology that divides the feature regions of different images. It includes several modules such as computer signal processing, image analysis, image fusion, segmentation, and recombination. The type, size, range, shape, and other information of the target are displayed in the figure in the form of division, and the final inspector will get the most intuitive image morphology [9]. At present, there have been research projects on applying tissue classification algorithm to the research of lung cancer, and there are very few research projects corresponding to cervical cancer. Therefore, the characteristic wavelength of whether the lesion occurs were adopted in this study, and the tissue classification algorithm-assisted multispectral imaging technology was applied to the screening and diagnosis of cervical cancer patients, so as to realize the early screening and discrimination of cervical cancer, providing theoretical reference for clinically rapid and efficient screening of cervical cancer.

## 2. Methods

### 2.1. Research Objects

In this study, 50 patients with suspected cervical cancer from October 2019 to October 2020 in the hospital were selected as the research objects. They were between 25 and 55 years old, with an average age of 40.2 ± 5.3 years.

The inclusion criteria were defined as follows: patients who were between 25 and 55 years old; patients with no pregnancy and no sexual history during the experimental study; patients with no symptoms of reproductive tract infections or bleeding; and patients without vagina operations such as lavage.

The exclusion criteria were defined as follows: patients with reproductive tract co-infected diseases or vaginal bleeding; women during pregnancy and menstrual period; patients who underwent cervical resection or took drugs to wash and treat the cervix within 48 hours; patients with mental or consciousness disorder and poor compliance; and patients who were allergic to alcohol.

All patients in this study and their authorized persons had signed the informed consent forms, and the study had been approved by the Medical Ethics Committee of the hospital.

### 2.2. Principle of Multispectral Imaging for Cervical Tissue Examination

The micro-snapshot narrowband multispectral imaging system was adopted in this study. Three narrowband multispectral images of 50 patients' cervical tissues were collected under conventional white light waveband, narrowband green light waveband, and narrowband blue light waveband, with the number of acquisition frames of about 25 fps. The specific details are shown in Figure 1.

### 2.3. Multiband Image Fusion

Before the organization algorithm, the multispectral image was firstly fused to eliminate the influence of factors such as different wavebands, degree of filtering, and conversion rate with different wavebands [9]. In this study, contrast was used to measure image clarity, and the below equation is taken as the calculation standard:

(1) $$\begin{array}{c} \mathrm{Contrast}=\sum_{\delta }\delta {\left(i,j\right)}^{2}p_{\delta }\left(i,j\right). \end{array}$$

In (1), *δ(i,j)* *=* *|i* − *j|* represents the difference in gray value between two adjacent image elements and *p*_*δ*_*(i,j)* refers to the distribution probability of two image elements when the gray value between the two adjacent image elements was *δ*.

### 2.4. Multispectral Fusion Image Combined with Tissue Classification Algorithm

Due to the difference in the contrast of the multiband spectrum fusion image between the uninfected cervical tissue and the diseased cervical tissue, the gray value of the lesion area is generally slightly smaller than that of the normal tissue [10]. Therefore, the tissue classification algorithm was used to classify the spectra of different tissues in this study. The tissue classification algorithm is to use the band characteristics or spatial characteristics of the multispectral image as the boundary between normal and diseased, so that the elements on the spectrum are divided into different levels or categories, thereby realizing alternative subjective analysis [11]. The tissue classification algorithm used in this study was mainly to adopt the K-value clustering algorithm to summarize and analyze the physiological and pathological regional features of the cervical cancer site and then apply the corresponding regional features to analyze the cervical tissues of 50 patients with no lesions. The second step was to convert a monochrome black and white image into a distribution image of a given color. The algorithm principle is shown in Figure 2. The K-means clustering (KMC) algorithm was adopted to divide the lesion area and the nonlesion area, and then a single gray-scale image was stored into a multicolor image that can be intuitively distinguished. On the one hand, it improved the precise identification of the target area on multispectral imaging and increased the feature discrimination of the image and the features that can be easily distinguished; on the other hand, it can also make the clinical imaging physicians more acceptable when judging the multispectral imaging map intuitively [12]. Therefore, after the KMC algorithm obtained the gray image, the most classic Bayer image color array format interpolation algorithm was used. In this study, the diseased cervical tissue was marked in red, and the normal cervical tissue was marked in green.

### 2.5. Evaluation Indicators for Tissue Classification Algorithm-Assisted Multispectral Image

In order not to be affected by subjective evaluation, a quantitative evaluation equation was adopted to evaluate the image quality, so as to evaluate the restored color images through quantitative indicators to improve the accuracy of image discrimination. The average gradient, SD, and image entropy were selected as the evaluation indicators to restore the image results. The results of this study were compared with the reported International Commission on Illumination (CIE) color reduction method [13]. In the below equations, *G* represents the average gradient, which was the average of the image gray value change rate and used to reflect the sharpness of the image; and the larger the *G*, the better the image; *SD* represents the dispersion of the pixels and the average value in the image. Generally, the larger the SD value, the higher the image pixels and the better the quality; *H* is the image entropy, which represents the characteristics of all gray values of each image. The larger the value of *G*, the more average information the image contains and the better the image quality.

(2) $$\begin{array}{c} G=\frac{1}{M\times N}\sum_{i=1}^{M}\sum_{j=1}^{N}\sqrt{\frac{{\Delta f/\Delta x}^{2}+{\Delta f/\Delta y}^{2}}{2}}, \end{array}$$

(3) $$\begin{array}{c} \text{SD}=\sqrt{\frac{1}{M\times N}\sum_{i=1}^{M}\sum_{j=1}^{N}{\left(p_{i,j}-\bar{x}\right)}^{2}}, \end{array}$$

(4) $$\begin{array}{c} H=-\sum_{i=0}^{n-1}p_{i}\log_{2}p_{i}. \end{array}$$

In (2) above, *M* × *N* represents the size of the image; *i* and *j* represent the pixel value of an element in the *i*-th row and *j*-th column, respectively; Δ*f*/Δ*x* is the image on the *X* axis (horizontal direction); and Δ*f*/Δ*y* is the gradient of the image on the *Y* axis (vertical direction). In (3), *P*_*i,j*_ represents the pixel value of the *i-*th row and *j* column; and $\bar{x}$ represents the average value of the image. In the above equation (4), *n* − 1 represents the *n* − 1 gray levels of the image, and *p*_*i*_ refers to the probability of occurrence of the *i*-th gray value.

### 2.6. Indicators for Combination of Algorithm and Clinical Examination

The aforementioned tissue classification algorithm combined with multispectral imaging was used to systematically examine the cervical cancers of 50 patients. In order to prevent infection, in all patients were used disposable operating tools during the examination, and experienced imaging physicians and gynecologists perform biopsy sampling, detection, image collection, and analysis of results. At least 3 test points were collected for each patient. Sensitivity and specificity were selected as the indicators of the algorithm in clinical multispectral imaging.

(5) $$\begin{array}{c} \mathrm{Se}=\frac{A}{A+C}\times 100\%. \end{array}$$

(6) $$\begin{array}{c} \mathrm{Sp}=\frac{B}{C+B}\times 100\%. \end{array}$$

In equations (5) and (6) above, *Se* and *Sp* refer to the sensitivity and specificity, respectively; *A* means that the results of the disease examination and the algorithm check of this research were both positive (with disease); *B* means that the results of the disease examination and the algorithm check of this study were both negative (no disease); *C* means that the result of the disease examination was positive and the result of algorithm adopted in this study was negative; and *D* means that the side-by-side result was negative and the result of this algorithm was positive.

## 3. Results

### 3.1. Multiband Image Fusion Results

After all the cervical tissues were preprocessed, the images were fused and processed according to whether different cervical tissues had different characteristic bands and response to light. It was found that there was a great difference between the fused spectral image 3(b) and the image 3(a) without lesions. At the same time, it was found that the contrast of the fused spectral image was 0.7549, which was also higher than the contrast of 0.4716 after the fusion, showing statistical difference (*P* < 0.05). It indicated that the separation of the fused image was improved and the image was clearer, as shown in Figures 3 and 4.

### 3.2. Algorithm-Assisted Spectral Image Results

The histological algorithm and multispectral image were combined to perform K-means unsupervised classification processing and color restoration technology on the collected cervical tissue.  Figure 5(a) shows the 3 detection points of the cervical tissue and whether there were lesions.  Figure 5(b) shows the multispectral image after fusion processing and the location of the detection points on the image.  Figure 5(c) shows the tissue classification algorithm-assisted fusion processing spectral cervical tissue and the results of segmentation in this image. The green mark in the figure is the area without lesions, while the red mark is the area with lesions. In the results of tissue classification diagnosis, Figure 5(c) is more intuitive than Figures 5(a) and 5(b) for whether the cervical tissue was cancerous or not and its scope, making it easier for clinicians to diagnose quickly.

### 3.3. Evaluation Indicators for Tissue Algorithm Image

The restored image was evaluated using three indicators. As given in Figure 6, the multispectral image average gradient, SD, and image entropy in this study based on the tissue classification algorithm were 2.0765, 65.2579, and 4.974, respectively, which were higher in contrast to the reported values (1.1777, 50.4657, and 3.9025, respectively), showing statistical difference (*P* < 0.05). It disclosed that the multispectral cervical tissue image based on the tissue classification algorithm was clearer, the segmentation of the lesion was clearer, and the overall quality of the image was better. Therefore, it could be applied in clinics to assist doctors in effectively completing the diagnosis of cervical cancer.

### 3.4. Results on Clinical Examination Indicators

To test the clinical performance of the tissue classification algorithm for cervical cancer tissue screening, the overall performance was evaluated by using two indicators (sensitivity and specificity). The multispectral image was compared with the tissue classification algorithm and the multispectral image without the algorithm. It was found (as illustrated in Figure 7) that the sensitivity and the specificity of the multispectral image with the tissue classification algorithm were 85.3% and 70.8%, respectively, both of which were larger than those of the images without the algorithm. Such results suggested that the use of tissue classification algorithm to assist multispectral imaging in screening cervical cancer showed higher accuracy and clinical application value.

## 4. Discussion

There are nearly 150,000 new cases of cervical cancer in China each year, and deaths due to cervical cancer account for nearly 20% of the female tumor deaths all over the world. The main cause of cervical cancer is that women are infected by human papillomavirus (HPV) [14]. Infection with high-risk HPV can cause abnormal cancer of the cervix and cause epithelial damage of the cervix. Women who are infected with high-risk HPV, without effective and timely treatment, will have a 10% chance of developing persistent HPV. Persistent HPV will continue to infect epithelial cells in the cervical tissue, causing heterogeneous proliferation of cervical epithelial cells, triggering cervical epithelial cancer, and greatly increasing the risk of eventually becoming cervical cancer [15]. Some researchers use HPV virus testing to screen cervical cancer to improve the screening and early diagnosis of cervical cancer. The detection method proposed by Digene has little specificity for HPV detection, the specificity for detecting all types of HPV viruses is not more than 10%, and the specificity for detecting high-risk HPV viruses that have been typed is only 30% [16]. Testing for HPV not only is low in specificity and produces unsatisfactory results but also causes physical and psychological distress to women. In recent years, some physicians have used multispectral imaging technology to assist in the screening of cervical cancer. Generally speaking, most new HPV infections do not cause symptoms or the disease can resolve spontaneously, but persistent infection with high-risk HPV (mainly types 16 and 18) may cause precancerous lesions. The high incidence of HPV infection is usually between 16 and 20 years old. It usually heals on its own but may also continue to be infected. If it is not treated in time, it may develop into cervical cancer after 10 to 20 years. Therefore, if cervical cancer can be detected early and treated early, most patients can be cured. Therefore, early screening and diagnosis of cervical cancer is of great significance for reducing the morbidity and mortality of patients. Cervical cancer screening begins with the introduction of Hirsch cytology test into the clinic as a routine screening item. At present, the early diagnosis and identification methods for cervical cancer have different shortcomings. Multispectral imaging examination, as a way of using the optical changes of cervical cancerous tissue, is noninvasive and effective in the screening of cervical cancer.

Multispectral imaging generally refers to a type of spectrum with a narrowband and high resolution and does not specifically refer to a certain spectrum. Its imaging principle is a spatial three-dimensional cube image formed by an optical image at a certain wavelength. Through the multispectral image, not only the image data of the research target at a certain wavelength can be obtained, which is used to obtain the two-dimensional morphological data of the research object, but also the spectral data of a certain wavelength in the three-dimensional space can be used to obtain the research object information contained within the space. Therefore, multispectral imaging technology has been applied to various aspects [17]. Image fusion is also an important point in multispectral imaging technology. The definition of multispectral image fusion is to combine all the characteristic information of the multispectral image at the same wavelength through a specific combination. Relying on their spatial correlation and complementarity, it finally gets a clearer and higher resolution image than the original image [18]. In this study, it was found that after the cervical tissues of all patients were processed, the spectral image after image fusion processing and the image 3(a) without lesions were combined according to the characteristic wavelength band of different cervical tissues and the response to light. In addition, the contrast of the fused multispectral image was 0.7549, which was also higher than the fused contrast of 0.4716, indicating that the separation of the fused image was improved and the image was clearer.

At present, artificial intelligence algorithms have been widely used in the medical field. For example, Dorta-Estremera uses deep learning algorithms to identify unbalanced error reports in medical data [19]. The tissue classification algorithm uses the band characteristics or spatial characteristics of the multispectral image to classify it as the boundary between unoccurring lesions and suspected lesions, so that the elements on the spectrum are divided into different levels or categories, thereby realizing alternative subjective analysis [20]. In this study, the tissue classification algorithm was applied to analyze the multispectral image of cervical tissue. Comparison of unfused and fused multispectral images showed that after the tissue classification algorithm was used to process the fused cervical tissue image, the area and the range of the cervical tissue in the image were more intuitive so that it was easier for doctors to quickly screen out cancerous lesions by color classification. In addition, the restored image was evaluated using three indicators. The result revealed that the multispectral image average gradient, SD, and image entropy in this study based on the tissue classification algorithm were 2.0765, 65.2579, and 4.974, respectively, which were higher in contrast to the reported values (1.1777, 50.4657, and 3.9025, respectively). It suggests that the multispectral cervical tissue image based on the tissue classification algorithm is clearer, the segmentation of the lesion is clearer, and the overall quality of the image is better.

With the application of optical imaging and computer algorithm technology in medical treatment in recent years, multispectral imaging technology can present high-definition and high-resolution imaging and lesion screening of cervical tissue. Studies have found that the sensitivity of multispectral imaging technology can reach nearly 96% and the specificity can reach nearly 56% [21]. In this study, the multispectral image of the tissue classification algorithm was compared with the multispectral image of the nonapplied algorithm. It was found that the sensitivity and specificity of the multispectral image with the tissue classification algorithm were 85.3% and 70.8%, respectively, which were higher than those of the image without the algorithm. It indicates that the use of tissue classification algorithm to assist multispectral imaging shows higher accuracy and higher clinical application value in screening of the cervical cancer.

## 5. Conclusion

Multispectral imaging assisted by tissue classification algorithm can effectively screen for cervical cancer and can quickly, efficiently, and safely segment the cervical tissue from the lesion area and the no-lesion area. The segmentation result was the same as the result of the physician's medical examination, showing that its clinical application value was high. This study could provide a new idea for the clinical application of tissue classification algorithm-assisted multispectral imaging technology in the early screening and diagnosis of cervical cancer. However, there were still some shortcomings in this study. The included sample size was small. To obtain more detailed results, more sample studies are needed in the future.

## Figures and Tables

**Figure 1:** Schematic diagram of multispectral imaging system.

**Figure 2:** The algorithm principle.

**Figure 3:** Processed images of normal tissue and fusion image: (a) image of the extracted cervical tissue (b) image for lesion area after multispectral fusion processing.

**Figure 4:** Contrast of two extracted images. *Note.*^*∗*^ means the difference was statistically great in contrast to the fusion image (*P* < 0.05).

**Figure 5:** Classification and diagnosis results of tissues: (a) the 3 detection points of cervical tissue and whether there were lesions; (b) the multispectral image after fusion processing and the position of the detection points on the image; and (c) the tissue classification algorithm-assisted fusion processing spectral cervical tissue and the result of the segmentation.

**Figure 6:** Comparison on evaluation indicators of restored color images: (a) the average gradient of the image; (b) the standard deviation of the image; and (c) the image entropy of the image. ^*∗*^Compared with the CIE algorithm, the difference was statistically significant (*P* < 0.05).

**Figure 7:** Comparison on sensitivity and specificity: (a) comparison results of sensitivity and (b) comparison results of specificity.

## Data Availability

The data used to support the findings of this study are available from the corresponding author upon request.
